RETRACTED

# Relationship between Investor Sentiment and Price Fluctuation of SSE 50ETF Options

**DOI:** 10.1155/2022/8992779

**Published:** 2022-06-29

**Authors:** Yang Wang, Yinjie Zhang, Yuwei Fu

**Affiliations:** China University of Mining and Technology-Beijing, Beijing 100083, China

## Abstract

In this paper, we have studied the December call-options contract of SSE 50ETF options to put forward the sentiment composite index of options by means of the principal component analysis and to explore the relationship between such index and the fluctuation taking place in option prices. The empirical study has shown that the investor sentiment is correlated with option prices, and option prices prove to be more sensitive to the sentiment, whereas the impact imposed by the sentiment of option investors on option prices is more significant.

## 1. Introduction

Options are critical financial derivatives in the modern financial market. On Feb. 9, 2015, the SSE 50ETF option was officially listed and traded on the Shanghai Stock Exchange, becoming the first standardized option traded on exchange and the first stock option officially opened to investors in China. Judging from the current circumstances, the options trading in China is just starting. In addition, the country's understanding of the system and market rules is still in its infancy, with numerous issues left to be studied and addressed. Therefore, the research on the market of stock options is utterly significant to the development of the current option market in China.

As a form of representation of the behavioral finance theory in the empirical research, the investor sentiment is a quantifiable indicator key to the theory. Therefore, we take the investor sentiment as the starting point of the research and take the most active option contracts among the call-options due in December 2019, the product of China's stock options trading market, and the Shanghai Stock Exchange 50EFT option, to explore the price of China's stock options based on investor sentiment regularity.

The main structure of the article is as follows: The first part is literature review which primarily elaborates on the research results of behavioral finance and investor sentiment. The second part explains the establishment method, process, and data selection adopted in the sentiment composite index of stock option investors. The third part provides the empirical analysis results and explanations. The last part sets out the research conclusions and specific recommendations.

We constructed a composite index of investor sentiment with principal component analysis and selected four indicators that can represent investor sentiment in China's stock options market: trading volume, put-subscription ratio, open interest, and range of rise and fall. In the empirical research part, through the linear regression, VAR model, and other empirical processes, the impact of investor sentiment on stock option price volatility is explored. We get conclusions that can reflect the real relationship between sentiment and price in China's stock options market in the analysis results of the model. The conclusion is that there is a positive correlation between investor sentiment and option prices, and option prices are more sensitive to sentiment, and the comprehensive index of option investor sentiment has a more significant impact on option prices.

RETRACTED

## 2. Literature Review

The theory of behavioral finance was put forward and became well known to scholars in the middle and late 1970s. It explains the fluctuations and phenomena experienced by financial markets by analyzing human behaviors and psychological motivations, which is the most critical achievement in the research of financial theories [1, 2]. Academically, behavioral finance theorists raise questions on the assumption of investors' complete rationality, accounting for the fact that their studies are more inclined to the psychological changes of investors [3, 4]. During its emergence and development, behavioral finance is inseparable from relevant theories such as prospect theory, *mental accounting* theory, conformity behavior theory, and overconfidence theory. The following are the important theories of the rise and development of behavioral finance:

First is prospect theory. Prospect theory is the theoretical cornerstone of the rise and development of behavioral finance. Prospect theory, also known as expectation theory, was proposed by economists Kahneman and Tversky [5]. The theory believes that investors' investment behaviors may have the risk of loss, and investors tend to be more inclined to take risks, but, in the process of gaining returns, they are converted into a risk-averse mental state. The existence of prospect theory provides a solid theoretical background and a new research direction for economists to study financial markets and prompts scholars to pay more attention to the changes of individual decision-making psychology and behavior in venture capital in the process of financial research.

Second is “psychological account” theory. The “psychological account” theory was first proposed in a paper published by the famous British behavioral finance scientist Richard Thaler in 1985. The existence of mental account is the reason for the irrational deviation of investor behavior. This theory provides behavioral finance more reasonable theoretical support.

RETRACTED

Third is herd behavior theory. Scholars Froot and Sharfstein (1992) proposed that, in the process of financial transactions, investors tend to obtain and refer to the information provided by others (simplified here). Therefore, they tend to observe the behavior of other investors and predict it. Therefore, this herd behavior is also an important breakthrough in the research and solution of behavioral finance.

Fourth is overconfidence theory. The overconfidence theory emphasizes that when investors show this state of overconfidence, the trading volume of securities will increase, thus affecting the efficiency of market operation. The overconfidence theory supplements and extends the behavioral finance theory to a certain extent and also provides a psychological basis for further explaining the market anomaly [6, 7].

The research on the influence of investor sentiment on option trading market mainly focuses on the explanation of investor sentiment on the fluctuation of option market and the enlightenment of investor sentiment on the correction of option pricing model. When studying the smile curve of option trading, scholar Han found that when investors tend to call a certain option target, the volatility curve of index option tends to be flat. This phenomenon is defined as the volatility smile curve, but this situation cannot be reasonably explained by the traditional option pricing model. However, investor sentiment can well explain the emergence of this anomaly [8–10]. In studying the impact of investor sentiment on option implied volatility, scholar SEO [11] found that when option investors show positive sentiment, risk neutrality can well explain the future volatility of options. Considering investor sentiment, the prediction results of option implied volatility are more in line with the actual market situation and more accurate [11]. Yan Liqiao [12] constructed the sentiment index based on the newly launched options in China and introduced the single-phase binary tree pricing model to draw the conclusion that there is a positive correlation between option sentiment and option price.

## 3. Establishment of Investor Sentiment Index and Selection of Data

In this paper, investor sentiment is considered to be a vital factor influencing the price of stock options. To explore the internal relationship between them, the most critical method for the researchers is to build an option sentiment index that can reflect the sentiment of investors in the stock option market [13–16]. Therefore, in this paper, we have selected the principal component analysis method to calculate the sentiment composite indexes, which can reflect the sentiment of the stock option market and enable us to explore this market [17–20].

RETRACTED

### 3.1. Index Selection

In this paper, researchers have referred to the previous practices of establishing indexes by domestic and foreign scholars while selecting sources of the indexes. With an in-depth understanding of the connotation of various variables and examination of the relationship between these variables with the investor sentiment and behavior, we have adopted the principal component analysis to analyze the trading volume, Put/Call, open interest, and change and to construct the option sentiment composite index based on the development status, characteristics, and data availability of China's stock option market [13, 20–22]. The use of principal component analysis to construct a comprehensive index of investor sentiment can more accurately describe the true sentiment of investors in the trading market, thus making the research results of investor sentiment and the closing trend of the options market more rigorous and scientific. Therefore, this paper adopts the principal component analysis method as the method of constructing the comprehensive sentiment index.

### 3.2. Data Selection

In this paper, we have studied the SSE 50ETF option trading to analyze how its price changes under the influence of investor sentiment. The SSE 50ETF option product that we have selected in this study is the 50ETF call option contract to be expired in December of 2019 (50ETF C. Dec.), mainly because December is the month of expiration for quarterly monthly contract. Among option contracts, the time span of quarterly contracts is the longest. While choosing the data of quarterly contracts as the research object, we are able to reduce the error caused by extremely limited samples, lack of data, and nonmarket factors as much as possible. In 2019, there were a total of 16 products of 50ETF C. Dec. Based on the average daily trading volume during the contract period as the benchmark of the active option contract, it is calculated that the 50ETF C. Dec. 3.00 contract is the most active among the 16 contracts (the meaning of 3.00 in the subscription contract is the exercise price at the expiration of the corresponding option contract). We have carried out an empirical analysis on 16 option contracts with December as delivery month. Due to the limitation of paper length, we have selected the 50ETF C. Dec. 3.00 contract as an example for further study. Relevant data are drawn from historical transaction data available in the Wind database.

### 3.3. Establishment of Investor Sentiment Composite Index

The principal component analysis method is used to select common factors from relevant indicators that can reflect investor sentiment, so that the extracted indicator becomes a comprehensive proxy variable that can represent investor sentiment. The method of investor sentiment indicator was first proposed by Baker and Wurgler [23], extracting the first principal component of the variables that can reflect investor sentiment as a comprehensive indicator of investor sentiment and conducting financial market research. By comparison, it is found that the use of principal component analysis to construct a comprehensive sentiment index representing investor sentiment has a better effect on financial market research than a single investor sentiment index. Domestic researchers have also adopted this method to construct a comprehensive index of investor sentiment. For example, Lin [24] used the principal component analysis method to analyze the return of IPO stocks, the turnover rate of A-share market, the discount of closed-end funds, and the initial public offering of stocks. The first component is extracted from the four proxy indicators of turnover rate as the investor sentiment index. The research results show that the comprehensive investor sentiment index constructed with the above indicators as proxy variables can objectively reflect the investor sentiment in China's financial market. In the research of this paper, the use of principal component analysis to construct a comprehensive indicator of investor sentiment can more accurately describe the real sentiment of investors in the trading market, so that the research results of exploring investor sentiment and options market closing trends are more rigorous and scientific. Therefore, this paper adopts the principal component analysis method as the method to construct the comprehensive sentiment index.

RETRACTED

Subsequent to the selection and primary treatment (standardization) of proxy indexes, we can establish the composite indexes. In this study, we comprehensively compare the research methods of previous scholars and finally choose principal component analysis to construct a comprehensive emotion index. The principle of principal component analysis is that deleting the interrelated variables among all the variables related to the research problem will reflect the redundant variables of repeated information. At the same time, new variables are established to reduce the number of variables as much as possible, reject the pairwise correlation of new variables, ensure the comprehensiveness of the new variables in reflecting the research problem, and ensure the existence of original information. In mathematical principle, a group of variables that may have correlation relationship are transformed into a group of linearly uncorrelated variables through orthogonal transformation, and the transformed variables are the main components. Therefore, after principal component analysis, the number of principal components can be determined and the expression of principal components can be established according to the correlation between proxy variables, so as to construct a comprehensive emotion index.

Using SPSS 20.0 software to reduce the dimension of 16 groups of proxy variables, the KMO statistics of the 16 groups of data are all above 0.5000, and the significance of the Bartlett test is all 0.000, indicating that the 16 groups of data can be reduced by principal component analysis. After principal component analysis, only the principal components whose eigenvalues are greater than 1 are extracted. After analysis of the 16 groups of data, only the first eigenvalue is greater than 1. The first factor can be extracted to explain most of the changes in the variables. All contracts in the study use the first principal component as an indicator of option sentiment. According to the eigenvector matrix obtained from the initial matrix, the weight occupied by each proxy index comprehensive sentiment index can be obtained. The source index data of 16 products are substitute into the corresponding comprehensive sentiment index calculation formula of each product, and the comprehensive sentiment index of option investors for each option product on each trading day is calculated.

After principal component analysis, we are able to extract a principal component, and then the sentiment composite index formula of 50ETF C. Dec. contract can be expressed as follows:

(1) $$\begin{array}{c} \text{FE}=0.466*\text{VOL}+\frac{0.259*P}{C}+0.466*\text{OI}+0.048*\text{CHG.} \end{array}$$

By substituting the source index data of the contract into the calculation formula, we can calculate the composite sentiment index of the option investor corresponding to each trading day of the option product. The option sentiment composite index is obtained as a time series. In addition, in order to verify the validity and stability of the option sentiment composite index calculated in this research, we have used the EViews 8.0 software to conduct the ADF test on the sentiment indexes that we obtained. The test results are specified as follows.

The results of the ADF test have shown that the sequence refuses the unit root hypothesis at a confidence level of less than 95%. Therefore, the sentiment composite index established in this paper is a stable sequence.

## 4. Empirical Study on Option Sentiment and Price Based on the VAR Model

### 4.1. Unit Root Test of Sequence

In this study, both sentiment sequence (E) and option price sequence (P) may not be stationary, whereas the stationary time sequence is the premise for performing Granger causality test and constructing the VAR model. Therefore, the stationary test of the two sequences is the primary task of subsequent research. In this paper, we have elaborated on the ADF test results of investor sentiment composite index and option price in terms of contracts. Each contract includes both sentiment sequence and price sequence. The ADF test results are set out as follows.

RETRACTED

Based on the test results shown in Tables 1-2, the investor sentiment composite index E and the option price P can reject the original hypothesis under the 5% test level, indicating that the two sequences are stable at the 95% confidence level. The Granger causality test and the VAR model can be directly carried out as follows.

### 4.2. Granger Causality Test

The Granger causality test is carried out mainly to test whether there is a causal relationship between varying variables, which relies on the null hypothesis. The null hypothesis refers to the hypothesis established in advance during the statistical test. When the null hypothesis holds, the relevant statistics should obey a known probability distribution. According to the principle of the Granger causality test, this test is used to analyze the sentiment composite index and option price sequence of option investors after stabilization. The test results are shown in Tables 3–5.

The results of the causality test in the tables have shown that, subsequent to the treatment of order 13, for the original hypothesis of the first line, the corresponding *P* value is 0.9914, which is far greater than the test level of 10%. Therefore, the original hypothesis cannot be rejected and we can draw the following conclusion; namely, Price P is not the Granger cause of the change in the sentiment variable E. Similarly, in the second line of hypothesis verification, the corresponding *P* value is 0.0264, which is less than the 5% statistical test level. Therefore, the original hypothesis can be rejected; namely, the sentiment variable sequence E is the Granger cause of the change in the option price sequence P, denoted as *E*⟶*P*.

After a large number of in-depth studies were conducted by both domestic and foreign scholars in recent years, economic and financial scholars have put forward views different from previous opinions on the Granger causality test; that is, the Granger causality test is used to verify the temporal order of statistical variables, but the test does not necessarily mean that there is a real causal relationship in economic principles. Therefore, instead of jumping to conclusions, this part of the Granger causality test results will be used as reference and validation. This paper will continue to build the VAR models to explore the specific impact relationship and mechanism between the two.

RETRACTED

### 4.3. Regression Results and Stationary Test of the VAR Model

In this paper, we have established the VAR model between the variable of the investor sentiment composite index and the option price, and, subsequent to the establishment of the model, we have determined its optimal lag period first.

According to the results of Table 6, in the first order, the values of the five principles of judgment are identified with; namely, the optimal lag order of the VAR model of the 50ETF C. Dec. 3.00 contract is one order, and then the VAR (1) model was established.

After determining the optimal lag period of the VAR model, we need to confirm the output results of the established VAR model, which are divided into two parts. The model includes the estimation of parameters of the established VAR model and the regression statistics of the model, which are set out as follows.

According to the model parameter estimates set out in Tables 7–9, the meaning represented by the small brackets is the standard deviation, and the meaning represented by the middle brackets is the t-test statistic. There are only two endogenous variables in the VAR model established in this paper, namely, the price variable (P) and the sentiment variable (E), which are ET and PT in this model, corresponding to two equations. Therefore, the estimated results of the VAR model obtained from the output results of the model are expressed as

(2) $$\begin{array}{c} \left[\begin{array}{c} \text{ET}\\ \text{PT} \end{array}\right]=\left[\begin{array}{c} 6932.773\\ 0.007036 \end{array}\right]+\left[\begin{array}{cc} 0.805858 & -234871.1\\ -5.01E-08 & 1.040818 \end{array}\right]{\left[\begin{array}{c} \text{ET}\\ \text{PT} \end{array}\right]}_{t-1}+\left[\begin{array}{cc} 0.138850 & 194412.9\\ 3.01E-08 & -0.107629 \end{array}\right]{\left[\begin{array}{c} \text{ET}\\ \text{PT} \end{array}\right]}_{t-2}. \end{array}$$

Once estimated results of the VAR model are obtained, it is necessary to check whether the VAR model proposed herein is stable. The AR root test results of the VAR model established in this paper are shown in Figure 1.

The output results of the stationary test on the model have shown that the points in the unit circle are the reciprocal of the root of the model's characteristic equation. Judging from the output test results, the points of the VAR model fall within the range of the circle, which proves that the VAR model established in this study on the relationship between option investor sentiment and option price is a stable model capable of being further analyzed and studied.

RETRACTED

### 4.4. Impulse Response Function

Since the impulse response function is an analytic method that responds to the shock of endogenous variables on the error term of the VAR model, we will analyze the impulse response of the established VAR model, option sentiment, and price in this paper. The results of the pulse response of the VAR model for 50ETF C. Dec. 3.00 contract are shown in the diagram as follows:

Judging from Figure 2 on the pulse response, we can conclude the following: First, the shock of option investor sentiment (ET) and option price (PT) on themselves shows a rapid downward trend in the early stage (i.e., the first and the second periods) and even experienced negative values. However, the price variable (PT) remains a flat state in the fourth period while approaching 0 after the fifth period. Furthermore, the sequence of sentiment variables (ET) tends to flatten in the sixth period while approaching zero after the seventh period in a gradually weakening fluctuation. The changes of the response of these two endogenous variables to their own shocks are characterized by a gradually weakening process before it is finally stabilized.

According to the diagram on the impulse response function of option price (PT) to option investor sentiment (ET), when the option price experienced a positive shock, the change of investor sentiment is 0 in the first period and slightly decreases in the second period. This is mainly because the change of price affects the acceptance information and investment decision-making of investors with periods characterized by a certain delay and a wait-and-see mentality. However, the price soon showed an upward trend and peaked in the third period; then the fluctuations flattened out and tended to zero in the fourth period. The vertical variation span of the whole response process is not very large, indicating that the change of option price will affect the investor sentiment with a lag effect. In addition, the effect is not long-term but responds with the change of price and tends to approach an equilibrium in the short term. Furthermore, though the effect exists, it remains rather weak.

According to diagram on the impulse response function of option investor sentiment (ET) to option price (PT), when a positive standard deviation shock from investor sentiment is received, the option price first decreases and then rises immediately and reaches a peak. Subsequently, the price begins to approach zero in the fourth period, indicating that the sentiment index has a positive impact on the market price in the short term. Based on such an impulse response mechanism, the response of option price to sentiment is also lagging. However, compared with the response of sentiment to price, the price is affected by sentiment during the second period, and the sentiment is affected during the third period. Therefore, the option price is more sensitive to the impact of option sentiment.

RETRACTED

### 4.5. Variance Decomposition

Variance decomposition is a method of studying the contribution of endogenous variables in the model to the variation of model prediction variance. The variance decomposition of 50ETF C. Dec. 3.00 contract is set out as follows with the results and analysis as shown in Table 9.

In Table 9, the column Period represents the prediction period of the standard deviation, and the column S.E. represents the standard deviation of variable prediction. In the variance decomposition of the sentiment composite index, the standard deviation of S.E. prediction of sentiment composite index in January amounts to 0.014285, and that of February amounts to 0.038995, which is slightly greater than the standard deviation of the prediction of January. This is because the prediction of February is affected by the uncertainty of prediction of January in terms of option price. While the number of prediction periods increases, the S.E. value of the sentiment composite index increases slowly. In the table on the variance decomposition results of the sentiment composite index, ET is listed as the percentage affected by itself in the prediction variance of the sentiment composite index, whereas PT is the percentage affected by option price during the prediction of the variance of the sentiment composite index, and the sum of both variables amounts to 100%.

Combining the variance decomposition results of the two variables, the price sequence contributes 3.357788% to the variance decomposition of the sentiment composite index in the tenth period, whereas the sentiment index contributes 4.942313% to the variance decomposition of the option price in the same period. In contrast, the contribution of sentiment to price variance decomposition is relatively higher, indicating that the explanatory rate of sentiment composite index to option price is higher than that of option price to sentiment composite index. Therefore, we can conclude that the sentiment composite index imposes a greater impact on the option price, corresponding to the result that sentiment is more sensitive to price changes in impulse response analysis.

## 5. Conclusions and Suggestions

In this paper, we have adopted the method of principal component analysis to establish the composite sentiment index of option sentiment, and we have set up a VAR model including both of these variables. In addition, we have tested the stability of the model and the Granger causality of the two variables. The results have shown that the VAR model established in this paper is a stable model with certain causal relationships among the variables. Based on the VAR model, we have conducted dynamic analysis in this study by means of impulse response and variance decomposition on the two variables and come to a more consistent conclusion; namely, the impact of option investor sentiment composite index on option price is more sensitive and significant. This conclusion is economically reasonable.

RETRACTED

The study is based on the relevant transaction data of China's stock option market, and we have explored the investor sentiment to provide suggestions and reference for the decision-making of investors in this market. The research of this paper can provide some reference and suggestions for investors in China's stock option market and help investors to have a deeper understanding of China's stock option market; at the same time, it is an in-depth exploration of China's stock option market, provides empirical basis for the impact mechanism of investors' behavior in China's stock option market, and is of great significance to the healthy and long-term development of China's stock option market.

According to the results of this paper and judging from the actual situation of China's stock option market, the following suggestions are provided from three aspects, that is, investors, market participants. and supervisors.

The stable operation of the stock option market is inseparable from the positive and optimal sentiment of the investors. In other words, it is necessary for the investors to stay constantly conscious in the option market and evaluate the fluctuations and changes of the stock option market in an objective and professional manner. In addition, the investors need to properly analyze the external information received in the option investment and cope with the fluctuation of the stock option market, since it is vital for the investors to make decisions carefully and maintain a positive and stable sentiment so as to ensure stable operation of the stock option market.

As a vital participant in the stock option market and a critical part of maintaining an active stock option market, listed companies play a pivotal role in the stock option market. In the development of the stock option market, it is essential for the investors to gain access to true and effective information so as to make better investment decisions. Listed companies should properly disclose information, so that the market can truly judge the value of the company, and these companies should also properly make pricing decisions so as to reduce the excessive fluctuation of investor sentiment caused by the lack of transparent information.

RETRACTED

As a guarantee for the sound operation of the stock option market, the government and relevant market supervision departments must play an effective role. First, policies and regulations must be formulated in accordance with the actual situation of the stock options market, and the government needs to ensure transparency and prevent investors from making irrational investment decisions, while minimizing the impact of policy risks on market operation. Second, the government needs to keep in check the excessive intervention of policies and regulations on the operation of the stock option market so as to ensure the effective play of market self-regulation function and to avoid the impact of excessive intervention on investors' investment behaviors and decision-making [20, 25–33].

## Figures and Tables

**Figure 1:** AR roots of the stationary test on the VAR model for 50ETF C Dec. 3.00 contract.

**Figure 2:** Results of the impulse response function of the VAR model for 50ETF C Dec. 3.00 contract.

**Table 1:** Description of sentiment indexes and prediction of relevant relationships.

Name of indexes	Symbols	Source of data	Category of data	Prediction of correlation with the established index
Trading volume	VOL	Wind financial database	Objective index	Positive correlation
Open interest	OI	Wind financial database	Objective index	Positive correlation
Put/Call	P/C	Wind financial database	Objective index	Negative correlation
Change	CHG	Wind financial database	Objective index	Positive correlation

**Table 2:** ADF test of option composite sentiment index.

Option composite sentiment index	ADF test value	1% confidence level	5% confidence level	10% confidence level	*P* value	Conclusion (%)
FE	−2.229979	−2.580065	−1.942910	−1.615334	0.0253	5

**Table 3:** Results of the stationary test on investor sentiment (E) for C. Dec. 3.00 contract.

		*t*-Statistic	Prob.
Augmented Dickey-Fuller test statistic		−2.229979	0.0253
Test critical values:	1% level	−2.580065	
	5% level	−1.942910	
	10% level	−1.615334	

**Table 4:** Results of option price (P) stationary test for C. Dec. 3.00 contract.

		*t*-Statistic	Prob.
Augmented Dickey-Fuller test statistic		−2.101656	0.0346
Test critical values:	1% level	−2.579139	
	5% level	−1.942781	
	10% level	−1.615416	

**Table 5:** Results of the causality test for 50ETF C. Dec. 3.00 contract.

Null hypothesis:	Obs	F-Statistic	Prob.
PT is not Granger cause of ET	143	0.40298	0.9914
ET is not Granger cause of PT		1.80365	0.0264

RETRACTED

**Table 6:** Selection results of the lag period of the VAR model for 50ETF C. Dec. 3.00 contract.

Lag	LogL	Lr	FPE	AIC	SC	HQ
0	−1720.650	NA	11626921	21.94459	21.98352	21.96040
1	−1368.613	690.6201	138033.5	17.51100	17.62780	17.55843
2	−1364.941	7.110500	138615.8	17.51517	17.70984	17.59423
3	−1363.223	3.283562	142714.6	17.54424	17.81677	17.65492
4	−1362.930	0.551723	149636.3	17.59147	17.94186	17.73377
5	−1361.170	3.273567	153999.5	17.62000	18.04826	17.79393
6	−1351.741	17.29676	143751.9	17.55084	18.05697	17.75640
7	−1349.938	3.260713	147893.2	17.57883	18.16283	17.81601
8	−1347.482	4.381125	150910.6	17.59849	18.26035	17.86730

^∗^indicates the lag order selected by the criterion.

**Table 7:** Parameter estimation results of the VAR model for 50ETF C. Dec. 3.00 contract.

	ET	PT
ET (−1)	0.805858	−5.01E−08
	(0.07852)	(4.4E−08)
	[10.2637]	[2.14268]

ET (−2)	0.138850	3.01E−08
	(0.07870)	(4.4E−08)
	[1.76422]	[2.68503]

PT (−1)	−234871.1	1.040818
	(143009.)	(0.07984)
	[−1.64235]	[13.0365]

PT (−2)	194412.9	−0.107629
	(140484.)	(0.07843)
	[2.38388]	[−1.97230]

C	6932.773	0.007036
	(6760.52)	(0.00377)
	[2.02548]	[1.86427]

**Table 8:** Regression results of the VAR model for 50ETF C. Dec. 3.00 contract.

*R*-squared	0.912465	0.923215
Adj. *R*-squared	0.910248	0.921271
Sum sq. resids	1.03E + 11	0.032242
S.E. equation	25587.67	0.014285
F-Statistic	411.7455	474.9213
Log likelihood	−1883.176	463.7639
Akaike information criterion (AIC)	23.16780	−5.629005
Schwarz criterion (SC)	23.26270	−5.534104
Mean dependent	45951.34	0.107621
S.D. dependent	85410.19	0.050911
Determinant resid. covariance (DOF adj.)		133368.4
Determinant resid. covariance		125311.8
Log likelihood		−1419.267
Akaike information criterion		17.53701
Schwarz criterion		17.72681

**Table 9:** Variance decomposition results of the VAR model for 50ETF C. Dec. 3.00 contract.

Variance decomposition of ET:				Variance decomposition of PT:			
Period	S.E.	ET	PT	Period	S.E.	ET	PT
1	0.014285	99.82165	0.198353	1	25587.67	0.000000	100.0000
2	0.020697	99.61725	0.382754	2	33121.21	1.734401	98.26560
3	0.025136	99.33774	0.662258	3	39161.99	2.436810	97.56319
4	0.028471	99.02586	0.974137	4	43961.46	2.965895	97.03410
5	0.031109	98.68700	1.313004	5	47977.84	3.388071	96.61193
6	0.033260	98.31996	1.680039	6	51411.69	3.754681	96.24532
7	0.035260	97.92806	2.071938	7	54396.57	4.085123	95.91488
8	0.036570	97.51510	2.484895	8	57021.53	4.389816	95.61018
9	0.037870	97.08515	2.914845	9	59350.60	4.674420	95.32558
10	0.038995	96.64221	3.357788	10	61431.58	4.942313	95.05769

## Data Availability

The datasets used and/or analyzed during this study are available from the corresponding author upon reasonable request.
